The article "Effect of Low-Frequency Electric Pulse Technique Combined with Carboprost Methylate Suppositories on Recovery of Gastrointestinal Function and Postoperative Complications of Patients with Scarred Uterus Undergoing Secondary Cesarean Section" was published in 2021. Journal: J Healthc Eng.

# Effect of Low-Frequency Electric Pulse Technique Combined with Carboprost Methylate Suppositories on Recovery of Gastrointestinal Function and Postoperative Complications of Patients with Scarred Uterus Undergoing Secondary Cesarean Section

**DOI:** 10.1155/2021/6143421

**Published:** 2021-11-24

**Authors:** Jinling Yan, Yongli Liu, Ruifen Jiao, Meixiang Li, Liqin Zhao

**Affiliations:** Department of Obstetrics, Shijiazhuang Obstetrics and Gynecology Hospital, Shijiazhuang 050000, Hebei Province, China

## Abstract

The study aims to explore the effect of low-frequency electric pulse technique combined with carboprost methylate suppositories on recovery of gastrointestinal function and postoperative complications of patients with scarred uterus undergoing secondary cesarean section (C-section). The clinical data of 120 patients with scarred uterus undergoing secondary C-section treated in our hospital from February 2019 to February 2020 were retrospectively analyzed, and the patients were equally divided into experimental and control groups according to their admission order, where each group included 60 patients. After the operation, patients in the control group received routine nursing and conducted breastfeeding, and carboprost methylate suppositories were used for postoperative hemostasis. Those in the experimental group received low-frequency electric pulse technique for comprehensive treatment to compare their coagulation function indicators, recovery of gastrointestinal function, incidence rates of postoperative complications, and involution of uterus. No significant between-group differences in patients' general information such as gestational weeks, gravidity, and number of times receiving C-section were observed (*P* > 0.05). Compared with the control group after the operation, patients in the experimental group obtained significantly better coagulation function indicators (*P* < 0.001) and presented better gastrointestinal function recovery (*P* < 0.001), significantly lower incidence rates of postpartum hemorrhage, retention of urine, deep venous thrombosis of lower limb, rupture of uterus, and endometrial cavity fluid (*P* < 0.05), and significantly better involution of uterus (*P* < 0.001). In conclusion, combining low-frequency electric pulse technique with carboprost methylate suppositories can lower the incidence rates of postoperative complications for patients with scarred uterus undergoing secondary C-section, improve their coagulation function, promote the recovery of gastrointestinal function, and present the desirable involution of uterus, which should be promoted in practice.

## 1. Introduction

A scarred uterus refers to a uterus that has undergone cesarean section (C-section) or intramural hysteromyoma cystectomy, and such uterine scar site is different from the surrounding normal myometrial wall, so it belongs to a high-risk pregnancy type [1]. Patients usually undergo C-section, the operation of removing the fetus and its appendages through laparotomy and cutting the uterus, when meeting the corresponding indications. With the continuous development of perinatology in China, the selection rate of C-section in the clinic has gradually increased [2, 3] because it can relieve long-term uterine contraction pain and production suffering. However, it is not an aseptic procedure, and, combined with the effects of anesthesia and surgical trauma, patients are prone to postoperative complications such as enteroplegia, ankylenteron, empty sagging in the lower abdomen, and postpartum hemorrhage [4, 5]. In addition, the slow uterine involution and prolonged duration of lochia caused by C-section also increase the difficulty of postpartum recovery. Compared with nonscarred uterus, the possibility of the previously mentioned complications in patients with scarred uterus undergoing secondary C-section is significantly increased [6]. A large number of studies show that scarred uterus is a risk factor for complications such as postpartum hemorrhage, which is the primary cause of postoperative death in patients undergoing C-section [7, 8]. Although the consensus of secondary vaginal trial delivery of scarred uterus has appeared in recent years, many patients with scarred uterus still prefer C-section [9], and therefore, rational application of drug treatment to reduce the incidence of postoperative complications is an important measure to guarantee the health of mothers and infants. At present, prostaglandin is the most commonly used hemostatic drug in clinic, and in addition to oxytocin, carboprost methylate suppositories can also contract uterine smooth muscle and have a preventive and therapeutic effect on postpartum hemorrhage that has been confirmed by international literature [10]. Not only that, carboprost methylate suppositories are able to stimulate the intestinal bladder smooth muscle and subsequently accelerate the recovery of gastrointestinal function of patients, which is beneficial to reduce the chance of abdominal distension and pain, so it has a significant efficacy in preventing postoperative complications in patients undergoing C-section.

The article "Effect of Low-Frequency Electric Pulse Technique Combined with Carboprost Methylate Suppositories on Recovery of Gastrointestinal Function and Postoperative Complications of Patients with Scarred Uterus Undergoing Secondary Cesarean Section" was published in 2021. Journal: J Healthc Eng.

On the basis of drug therapy, jointly adopting other rehabilitation techniques after C-section can accelerate the progress of uterine involution in patients and shorten the duration of lochia rubra [11]. Low-frequency electric pulse technology is a widely applied postpartum rehabilitation intervention in recent years, which is able to accelerate the pelvic floor blood circulation and promote uterine ligaments movement in patients through physical therapy. Some studies show that the low-frequency electric pulse instrument can also ensure unobstructed mammary gland, favoring the promotion of breast milk secretion [12]. As more and more patients with scarred uterus currently choose C-section, the combination of carboprost methylate suppositories and low-frequency electric pulse technique may not only reduce the complication rate and accelerate the postoperative recovery of patients but also lead to huge economic benefits with good market-based prospects.

Reviewing previous literature, the combination of carboprost methylate suppositories and low-frequency electric pulse technique is mainly adopted in patients undergoing C-section for the first time, and there are no studies on using the combination for patients with scarred uterus undergoing secondary C-section. A total of 120 patients were included in the study and divided into the control group and experimental group. The patients in the control group received the combination treatment of routine nursing, breastfeeding, and carboprost methylate suppositories, and those in the experimental group received the combination treatment of carboprost methylate suppositories and low-frequency electric pulse technique. It was found that patients in the experimental group presented significantly better comprehensive efficacy. The study contents were summarized as follows.

## 2. Data and Methods

### 2.1. Study Design

This was a retrospective analysis study conducted in our hospital from February 2019 to February 2020 to explore the effect of combining low-frequency electric pulse technique with carboprost methylate suppositories on recovery of gastrointestinal function and postoperative complications of patients with scarred uterus undergoing secondary C-section.

### 2.2. Recruitment of Study Objects

The clinical data of patients with scarred uterus undergoing secondary C-section treated in our hospital from February 2019 to February 2020 were retrospectively analyzed. Inclusion criteria were as follows: (1) the patients had a history of uterine surgery, and the results of pregnancy ultrasonography met the diagnostic criteria of scarred uterus in *Obstetrics and Gynecology* [13]; (2) the patients had clear indications of C-section or failed in trail delivery for scarred uterus; (3) the patients were cases of singleton pregnancy; (4) the patients were treated in our hospital throughout the entire process, and no situations such as death, transferring to another hospital, or discontinuation of treatment occurred. Exclusion criteria were as follows: (1) the patients could not communicate with others due to hearing disorders, language disorders, unconsciousness, or mental diseases; (2) the patients quit the treatment, died, changed the treatment regimen, or went missing in follow-up visits; (3) the patients were cases of multiple pregnancy; (4) the intrauterine growth was abnormal with the presence of severe eclampsia, placental adherence, or placenta praevia; (5) the patients had combined liver, kidney, heart and brain dysfunction, pelvic infection, coagulation disorders, or other severe pregnancy complications; (6) the patients had subarachnoid space tissue contraindication; (7) the patients had nipple abnormality; (8) the patients were allergic to the drugs involved in the study.

The article "Effect of Low-Frequency Electric Pulse Technique Combined with Carboprost Methylate Suppositories on Recovery of Gastrointestinal Function and Postoperative Complications of Patients with Scarred Uterus Undergoing Secondary Cesarean Section" was published in 2021. Journal: J Healthc Eng.

### 2.3. Steps

A total of 120 patients were included in the study and equally divided into experimental and control groups according to their admission order, where each group included 60 patients. On the day that the patients agreed to join the study, the study team collected their sociodemographic data and clinical performance data, and no statistical between-group differences in patients' general information were observed after analysis (*P* > 0.05) (see Table 1).

### 2.4. Moral Consideration

The study met the principles in the *World Medical Association Declaration of Helsinki* [14] and was approved by the review committee of the hospital ethics review organization. After recruitment, the study team explained the study purpose, meaning, contents, and confidentiality to the patients and asked the patients to sign the informed consent.

### 2.5. Criteria of Quitting the Experiment

If the patients had one of the following situations and the study team determined that they were not suitable for continuously accepting the experiment, their case records would be retained and not used for data analysis: (1) those who had adverse events or serious adverse events; (2) those with a condition worsening during the experiment; (3) those who had certain serious comorbidities or complications; (4) those who were unwilling to proceed with the clinical trial and demanded quitting.

### 2.6. Methods

After the operation, patients in the control group received routine nursing and conducted breastfeeding and were administered carboprost methylate suppositories to prevent postoperative hemorrhage. After delivery of the fetus, 20 U of oxytocin (manufactured: SPH No. 1 Biochemical & Pharmaceutical Co., Ltd.; NMPA approval no. H31020861) was mixed with 500 ml of lactated ringer solution (manufactured: Weifang Renkang Pharmaceutical Co., Ltd.; NMPA approval no. H20123165) and administered to the patients via an intravenous drip, and at the same time, the patients took 1 mg of carboprost methylate suppository (manufactured: Northeast Pharm Group Shenyang No. 1 Pharmaceutical Co., Ltd.; NMPA approval no. H10800007) via sublingual administration. The oxytocin was administered continuously from the day of operation to days one and two after the operation.

The article "Effect of Low-Frequency Electric Pulse Technique Combined with Carboprost Methylate Suppositories on Recovery of Gastrointestinal Function and Postoperative Complications of Patients with Scarred Uterus Undergoing Secondary Cesarean Section" was published in 2021. Journal: J Healthc Eng.

On this basis, the patients in the experimental group received the comprehensive treatment with low-frequency electric pulse technique, and the specific measures were as follows. (1) Administer uterus involution therapy. At one day after the operation, help the patients to take the supine position, set the pulse frequency of the low-frequency electric pulse instrument (manufactured: Qisheng (Shanghai) Medical Equipment Co., Ltd.; NMPA (I) 20143234403) to 833 Hz and the pulse width to 0.4 ms, adjust the pulse intensity to the degree that could be tolerable by patients, apply the coupling agent on the black side of the plate, place the plate on the sacrococcygeal region of the patients and the other two mammary gland plates under the breasts and fix with the abdominal binder, keep the two electrodes 4-5 cm from each other, use the low frequency gear, and switch on and press the start button of uterus involution therapy procedure. The therapy lasted 25 min and was administered twice daily and for six consecutive days. (2) For patients with less than 5 ml of breast milk volume three days after the operation, apply the coupling agent on the two special mammary gland masks and place them on the breasts to closely contact with the skin, fix with the abdominal binder, use the low frequency gear, switch on and press the start button of lactation therapy procedure, and gradually increase the intensity to enhance the stimulation. The therapy lasted 25 min and was administered twice daily and for six consecutive days.

### 2.7. Observation Criteria

#### 2.7.1. General Information

The general information extract form was established by the patients themselves, covering the inpatient number, name, age, gestational weeks, body weight of the fetus, newborn Apgar scores, history of C-section, number of C-section, history of intramural hysteromyoma cystectomy, size of gestation sac, gravidity, place of residence, monthly income, educational degree, and living habits.

#### 2.7.2. Coagulation Function Indicators

Before the operation (T_1_), 2 h after the operation (T_2_), and 24 h after the operation (T_4_), the patients' coagulation function indicators, including their activated partial thromboplastin time (APTT), prothrombin time (PT), fibrinogen content (Fib), and D-dimer (D-D), were measured with the automatic coagulation analyzer (German-imported Coatron1800, original kit; NMPA (I) 20132402724).

The article "Effect of Low-Frequency Electric Pulse Technique Combined with Carboprost Methylate Suppositories on Recovery of Gastrointestinal Function and Postoperative Complications of Patients with Scarred Uterus Undergoing Secondary Cesarean Section" was published in 2021. Journal: J Healthc Eng.

#### 2.7.3. Recovery of Gastrointestinal Function

After the operation, the patients' bowel sound recovery time, anal exhaust time, first defecation time, and incidence rate of abdominal distention were recorded. Every 2 h, the study team listened to the patients' bowel sound with the stethoscope at the left upper part, left lower part, right upper part, and right lower part of their abdomen for 2 min each, and if the bowel sound could be heard at two areas and the frequency was more than four times per second, it was regarded as bowel sound recovery.

#### 2.7.4. Incidence Rates of Postoperative Complications

The postoperative complications included postpartum hemorrhage, retention of urine, deep venous thrombosis of lower limb, rupture of uterus, and pelvic adhesion, and the number of patients with such complications in each group was recorded.

#### 2.7.5. Involution of Uterus

The patients took the spine position (or lateral recumbent position if necessary). The frequency of convex probe of the color doppler ultrasonography (GE Healthcare Voluson P6; NMPA (I) 20152062178) was set to 3.5–5 MHz. Uunder the condition that the patients' bladders were nearly full of urine, their uterine height at postoperative 12 h (T_3_), 24 h (T_4_) and 72 h (T_5_) and the sum of the three uterine diameters and size of uterus at postoperative days 5 and 42 were observed. At the same time, amount and duration of lochia rubra were recorded.

### 2.8. Statistical Processing

In this study, the data processing software was SPSS20.0. The picture drawing software was GraphPad Prism 7 (GraphPad Software, San Diego, USA). The included items were enumeration data and measurement data. The used methods were *X*^2^ test and *t*-test, and differences were considered statistically significant at *P* < 0.05.

## 3. Results

### 3.1. Comparison of Patients' General Information

No statistical between-group differences in the patients' gestational weeks, gravidity, number of times receiving C-section, and other general information were observed (*P* > 0.05) (see Table 1).

### 3.2. Comparison of Patients' Coagulation Function Indicators

The postoperative coagulation function indicators were significantly better in the experimental group than in the control group (*P* < 0.001) (see Figure 1).

In Figure 1, the horizontal axes from the left to right indicated T_1_, T_2_, and T_4_, the lines with dots indicated the experimental group, the lines with blocks indicated the control group, and # denoted *P* < 0.001. Figure 1(a) shows APTT. At T_1_, no statistical between-group difference in APTT was observed (32.68 ± 2.12 vs. 32.78 ± 2.13, *P* > 0.05); and at T_2_ and T_4_, the APTT was significantly lower in the experimental group than in the control group (20.65 ± 2.15 vs. 24.68 ± 2.32, 23.12 ± 2.65 vs. 26.98 ± 2.87, *P* < 0.001). Figure 1(b) shows PT. At T_1_, no statistical between-group difference in PT was observed (14.22 ± 0.35 vs. 14.26 ± 0.36, *P* > 0.05); and at T_2_ and T_4_, the PT was significantly lower in the experimental group than in the control group (8.62 ± 0.26 vs. 10.23 ± 0.57, 10.89 ± 0.36 vs. 13.14 ± 0.68, *P* < 0.001). Figure 1(c) shows Fib. At T_1_, no statistical between-group difference in Fib was observed (2.45 ± 0.36 vs. 2.48 ± 0.35, *P* > 0.05); and at T_2_ and T_4_, the Fib was significantly higher in the experimental group than in the control group (2.05 ± 0.30 vs. 1.74 ± 0.35, 3.68 ± 0.41 vs. 3.23 ± 0.56, *P* < 0.001). Figure 1(d) shows D-D. At T_1_, no statistical between-group difference in D-D was observed (2.15 ± 0.35 vs. 2.12 ± 0.32, *P* > 0.05); and at T_2_ and T_4_, the D-D was significantly lower in the experimental group than in the control group (2.64 ± 0.35 vs. 4.15 ± 0.57, 3.12 ± 0.69 vs. 3.75 ± 0.68, *P* < 0.001).

The article "Effect of Low-Frequency Electric Pulse Technique Combined with Carboprost Methylate Suppositories on Recovery of Gastrointestinal Function and Postoperative Complications of Patients with Scarred Uterus Undergoing Secondary Cesarean Section" was published in 2021. Journal: J Healthc Eng.

### 3.3. Comparison of Patients' Gastrointestinal Function Recovery

The postoperative gastrointestinal function recovery was remarkably better in the experimental group than in the control group (*P* < 0.001) (see Figure 2).

In Figure 2, the horizontal axes from the left to right indicated the experimental group and the control group, and # means *P* < 0.05. Figure 2(a) shows the bowel sound recovery time, which was remarkably shorter in the experimental group than in the control group (8.11 ± 1.23 vs. 13.35 ± 2.10, *P* < 0.001). Figure 2(b) shows the anal exhaust time, which was remarkably shorter in the experimental group than in the control group (15.41 ± 2.35 vs. 26.78 ± 3.50, *P* < 0.001). Figure 2(c) shows the time of first defecation, which was remarkably shorter in the experimental group than in the control group (33.58 ± 5.68 vs. 53.57 ± 6.98, *P* < 0.001). Figure 2(d) shows the incidence rate of bloating, which was remarkably lower in the experimental group than in the control group (2 vs. 15, *P* < 0.05).

### 3.4. Comparison of Incidence Rates of Postoperative Complications

The incidence rates of postpartum hemorrhage, retention of urine, deep venous thrombosis of lower limb, rupture of uterus, and endometrial cavity fluid were greatly lower in the experimental group than in the control group (*P* < 0.05) (see Table 2).

### 3.5. Comparison of Involution of Uterus

The postoperative uterus involution was remarkably better in the experimental group than in the control group (*P* < 0.001) (see Figures 3 and 4).

The article "Effect of Low-Frequency Electric Pulse Technique Combined with Carboprost Methylate Suppositories on Recovery of Gastrointestinal Function and Postoperative Complications of Patients with Scarred Uterus Undergoing Secondary Cesarean Section" was published in 2021. Journal: J Healthc Eng.

Figure 3(a) shows the uterine height. The horizontal axis from the left to right indicated T_3_, T_4_, and T_5_, and the uterine height at the three time points was significantly lower in the experimental group than in the control group (5.12 ± 1.23 vs. 6.54 ± 1.52, 10.68 ± 1.54 vs. 12.98 ± 1.68, 8.45 ± 1.26 vs. 11.20 ± 1.65, *P* < 0.001). Figure 3(b) shows the sum of the three uterine diameters. The horizontal axis from left to right indicated postoperative days 5 and 42, and the sums of the three uterine diameters at the two time points were significantly lower in the experimental group than in the control group (32.98 ± 3.65 vs. 36.11 ± 3.54, 15.98 ± 2.65 vs. 17.98 ± 2.40, *P* < 0.001). Figure 3(c) shows the size of uterus. The horizontal axis from the left to right indicated postoperative days 5 and 42, and the size of uterus at the two time points was significantly smaller in the experimental group than in the control group (26.12 ± 1.21 vs. 33.58 ± 3.65, 17.65 ± 1.65 vs. 19.23 ± 1.68, *P* < 0.001).

In Figure 4, the horizontal axes from the left to right indicated the experimental group and the control group, and # means *P* < 0.001. Figure 4(a) shows the amount of lochia rubra, which was significantly lower in the experimental group than in the control group (162.98 ± 24.65 vs. 196.98 ± 32.65, *P* < 0.001). Figure 4(b) shows the duration of lochia rubra, which was significantly shorter in the experimental group than in the control group (14.55 ± 2.35 vs. 21.56 ± 3.65, *P* < 0.001).

## 4. Discussion

C-section refers to the operation for women whose gestation time is more than 28 weeks to remove the fetus and its appendages through laparotomy and cutting the uterus. The operation rate of C-section specified by the World Health Organization is less than 15%, but with the continuous progress of perinatology, it is increasing year by year worldwide, which is about 20% in European and American countries and more than 30% in China [15–17]. C-section can reduce the pain caused by contractions and delivery and is beneficial to protect the safety of the fetus due to the short operation time, so its operation rate is difficult to reduce in the clinic. Therefore, medical intervention and other methods must be taken to accelerate the uterine involution process and reduce the duration of lochia. With the implementation of China's policy on allowing families to have two children, the operation rate of C-section has been further improved [18], and so is the rate of getting pregnant with a scarred uterus. However, compared with the healthy individual, patients with scarred uterus have endometrial defects, destroyed uterine tissue integrity, and reduced contraction ability, which, combined with the organism damage caused by C-section, they are highly prone to postpartum hemorrhage due to uterine inertia, and their chances of developing complications such as postpartum infection and poor incision healing are increased. To improve the uterine contraction function of patients with scarred uterus, oxytocin therapy is often used clinically, which can reach the peak concentration after intravenous infusion for 3 min, with rapid effect and desirable safety. However, oxytocin has a short half-life and the maintenance time of drug effect is less than 1 h, which only has mild effect for patients with a scarred uterus who have severe uterine inertia [19], so applying oxytocin alone does not present an optimal result. In addition to oxytocin, prostaglandin drugs can also regulate somatic cell activity, stimulate uterine smooth muscle and accelerate contractions, presenting excitatory effects at all stages of pregnancy. Studies have shown that, as a common prostaglandin, carboprost methylate suppository can accelerate platelet aggregation and promote uterine smooth muscle contraction [20, 21], so the coagulation function indicators of both groups were improved, and the postpartum hemorrhage rate of patients was 10.8%, which was significantly lower than the general level.

The article "Effect of Low-Frequency Electric Pulse Technique Combined with Carboprost Methylate Suppositories on Recovery of Gastrointestinal Function and Postoperative Complications of Patients with Scarred Uterus Undergoing Secondary Cesarean Section" was published in 2021. Journal: J Healthc Eng.

Other than preventing postpartum hemorrhage, carboprost methylate suppository also regulates the gastrointestinal function. Patients undergoing C-section are prone to postoperative bowel paralysis symptoms such as abdominal distension and pain due to the influence of anesthesia and surgical trauma, and improving gastrointestinal function as early as possible can reduce the chance of occurrence of intestinal adhesion [22]. Therefore, restoring gastrointestinal function is the focus of treatment for patients with scarred uterus undergoing secondary C-section. The study by scholars Vimercati et al. showed that patients undergoing C-section and accepting carboprost methylate suppositories had significantly shorter bowel sound recovery time and anal exhaust more time than those in the control group (*P* < 0.001) and presented lower incidence rate of abdominal distension [23], which was similar to the results of this study. This demonstrates that carboprost methylate suppositories could directly act on the smooth muscles of intestinal tract and bladder and make them contract, thereby promoting the postoperative recovery of patients' gastrointestinal function and bladder function. Compared with the control group, the patients in the experimental group had more desirable gastrointestinal function, which might be closely related to the application of low-frequency electric pulse technique. Such technique can act on the sacrococcygeal region of puerpera, accelerate the pelvic floor blood circulation, and enhance the local water absorption rate, so that pelvic floor muscle contraction ability is promoted and fascial tension is elevated, which can drive the movement of uterine ligaments of patients to accelerate their uterine involution [24]. C-section requires cutting the uterine muscle bundles and cutting off the intramural vessels, so the blood supply in patients is affected even after suturing. In addition, due to the patient's prolonged bed rest after surgery and the high amount of postpartum blood loss, their pelvic floor muscle tone recovered slowly, which further affected the uterine contraction, so it was important to accelerate the postoperative uterine involution. In the study by scholars Gromis et al., it was shown that, at postoperative days 5 and 42, the size of uterus of patients undergoing C-section who accepted the low-frequency electric pulse treatment was 25.37 ± 1.28 and 16.73 ± 1.03, respectively [25], indicating that such treatment could accelerate the involution of uterus. In this study, after applying the low-frequency electric pulse treatment, patients in the experimental group had significantly better involution of uterus (*P* < 0.001), shorter duration of lochia, and significantly lower incidence rates of retention of urine, deep venous thrombosis of lower limb, rupture of uterus, and endometrial cavity fluid than the control group (*P* < 0.05), proving that combining carboprost methylate suppositories with low-frequency electric pulse technique had a more desirable and comprehensive effect.

The article "Effect of Low-Frequency Electric Pulse Technique Combined with Carboprost Methylate Suppositories on Recovery of Gastrointestinal Function and Postoperative Complications of Patients with Scarred Uterus Undergoing Secondary Cesarean Section" was published in 2021. Journal: J Healthc Eng.

## 5. Conclusion

To sum up, combining carboprost methylate suppositories with low-frequency electric pulse technique can reduce the complication rates in patients with scarred uterus undergoing secondary C-section, improve their coagulation function, accelerate the recovery of gastrointestinal function, and present a more desirable involution of uterus, which should be promoted in practice.

## Figures and Tables

**Figure 1:** Comparison of patients' coagulation function indicators ($\bar{x}\pm s$).

**Figure 2:** Comparison of patients' gastrointestinal function recovery.

**Figure 3:** Comparison of involution of uterus ($\bar{x}\pm s$). ^#^*P* < 0.001.

**Figure 4:** Comparison of postoperative lochia ($\bar{x}\pm s$).

**Table 1:** Comparison of patients' general information.

Group	Experimental (*n*=60)	Control (*n*=60)	*X* ^2^/*t*	*P*
Age (years)				
Range	25–38	24–38		
Mean age	30.25 ± 2.35	30.36 ± 2.41	0.253	0.801
Gestational weeks	38.65 ± 1.22	38.54 ± 1.23	0.492	0.624
Body weight of the fetus (g)	3456.82 ± 310.57	3458.98 ± 324.68	0.037	0.970
Newborn Apgar scores	9.14 ± 0.65	9.16 ± 0.57	0.179	0.858
History of C-section	48	46		
Number of times receiving C-section (times)	1.65 ± 0.48	1.70 ± 0.46	0.583	0.561
History of intramural hysteromyoma cystectomy	12	14		
Size of gestation sac (mm)	20.11 ± 2.10	20.08 ± 2.15	0.077	0.939
Gravidity (times)	2.89 ± 0.35	2.84 ± 0.30	0.840	0.403
Place of residence			0.036	0.850
Urban area	38	37		
Rural area	22	23		
Monthly income (yuan)			0.033	0.855
≥4000	28	29		
<4000	32	31		
Living habit				
Smoking history	15	16	0.044	0.835
Drinking history	18	17	0.040	0.841
Educational degree			0.034	0.855
Senior high school and below	28	27		
College and above	32	33		

**Table 2:** Comparison of incidence rates of postoperative complications (*n* (%)).

Group	Experimental (*n* = 60)	Control (*n* = 60)	*X* ^2^	*P*
Postpartum hemorrhage	3 (5.0)	10 (16.7)	4.227	0.040
Retention of urine	1 (3.3)	7 (11.7)	4.821	0.028
Constipation	1 (3.3)	6 (10.0)	3.793	0.051
Deep venous thrombosis of lower limb	0 (0.0)	7 (11.7)	7.434	0.006
Rupture of uterus	1 (3.3)	8 (13.3)	5.886	0.015
Pelvic adhesion	1 (3.3)	6 (10.0)	3.793	0.051
Endometrial cavity fluid	0 (3.3)	6 (10.0)	6.316	0.012

## Data Availability

The datasets used and/or analyzed during the current study are available from the corresponding author on reasonable request.
